The article "GSK1904529A, an insulin-like growth factor-1 receptor inhibitor, inhibits glioma tumor growth, induces apoptosis and inhibits migration" was published in 2015. Journal: Mol Med Rep.

# GSK1904529A, an insulin-like growth factor-1 receptor inhibitor, inhibits glioma tumor growth, induces apoptosis and inhibits migration

**DOI:** 10.3892/mmr.2015.3869

**Published:** 2015-05-28

**Authors:** QIANG ZHOU, JUNXIA ZHANG, QINYING CUI, XIAODONG LI, GE GAO, YANFEN WANG, YUPING XU, XIAOQUN GAO

**Affiliations:** 1 Department of Pathology, Children's Hospital of Zhengzhou, Zhengzhou, Henan 450052, P.R. China; 2 Department of Anatomy, Basic Medical College, Zhengzhou University, Zhengzhou, Henan 450001, P.R. China; 3 Department of Ophthalmology, People's Hospital of Zhengzhou, Zhengzhou, Henan 450012, P.R. China; 4 Department of Physiology, Basic Medical College, Zhengzhou University, Zhengzhou, Henan 450001, P.R. China; 5 Department of Dermatology, Henan Provincial People's Hospital, Zhengzhou, Henan 450003, P.R. China

**Keywords:** glioma, insulin-like growth factor I receptor, GSK1904529A, cell viability, apoptosis, migration, tumor growth

## Abstract

Malignant gliomas are the most common type of primary malignancy of the central nervous system, with a poor prognosis. The therapeutic options for malignant gliomas are limited and far from satisfactory, and novel treatment strategies are urgently required to improve the outcome of the disease. Insulin-like growth factor (IGF)/IGF-1 receptor (IGF-1R) signaling pathway regulates cell proliferation, motility and survival. The dysregulation of this signaling pathway has been implicated in the development of malignant gliomas. In the present study, GSK1904529A, a small molecule inhibitor of IGF-1R, suppressed glioma cell viability, induced glioma cell apoptosis and inhibited glioma cell migration *in vitro*. In addition, GSK1904529A inhibited glioma tumor growth and induced tumor cell apoptosis *in vivo*. In conclusion, the results of the present study suggested GSK1904529A as a promising agent for the treatment of malignant glioma.

## Introduction

Gliomas are the most common type of primary brain tumor in humans, accounting for >80% of all brain malignancies (1). Gliomas are classified into astrocytomas (Grade I–IV), oligo-dendrogliomas (Grade II and III), ependymomas (Grade I–III) and mixed oligo-astrocytomas (Grade II and III), according to the World Health Organization (1,2). Glioblastoma, also termed glioblastoma multiforme, is a Grade IV astrocytoma, which is the most aggressive form of glioma, and accounts for ~60–70% of all malignant gliomas worldwide (1,3). The prognosis for patients diagnosed with glioblastoma is particularly poor, with 1-year and 5-year survival rates at ~36% and 5%, respectively (1,4). Current treatments for malignant gliomas include maximal surgical resection whenever possible, radiotherapy and chemotherapy, however, no significant improvements in survival rates have been achieved (5) and there remains urgent requirement for the identification of novel molecular targets and therapies.

The article "GSK1904529A, an insulin-like growth factor-1 receptor inhibitor, inhibits glioma tumor growth, induces apoptosis and inhibits migration" was published in 2015. Journal: Mol Med Rep.

Insulin-like growth factor I receptor (IGF-1R) is a tyrosine kinase receptor, which binds to IGF1 and IGF2. Upon ligand binding, IGF-1R activates the Ras/mitogen-activated protein kinase (MAPK) and phosphoinositide 3-kinase (PI3K)/AKT signaling pathways and regulates cell proliferation and survival (6). The IGF/IGF-1R signaling axis has been implicated in the development of several types of solid tumor by promoting the growth and survival of malignant cells (7–9). Previous studies have demonstrated that this pathway is also involved in the development of gliomas (10–14). Therefore, the IGF/IGF-1R signaling pathway may be a potential target for the treatment of glioma. GSK1904529A is a small molecule inhibitor of IGF-1R and has been demonstrated to inhibit the proliferation of several tumor cells by inhibiting receptor phosphorylation and downstream signaling (15). In the present study, the antitumor activity of GSK1904529A in glioma was assessed. Evaluation of the effects of GSK1904529A on the viability, apoptosis and migration of glioma cells may elucidate its effect on glioma tumor growth *in vivo* and determine its potential for the treatment of glioma.

## Materials and methods

### Reagents and cells

GSK1904529A was purchased from GlaxoSmithKline (Research Triangle Park, NC, USA), and was dissolved in dimethyl sulfoxide for *in vitro* investigation or 20% sulfobutylether-β-cyclodextrin for *in vivo* investigation.

The U87MG cells were purchased from American Type Culture Collection (Manassas, VA, USA) and were maintained in complete Dulbecco's modified Eagle's medium (DMEM), supplemented with 10% fetal bovine serum.

### Cell viability assay

The cells (1,000 cells/well) were seeded into 96-well plates in triplicate and incubated overnight at 37°C. The cells were subsequently treated with GSK1904529A at the indicated concentrations for 24, 48 or 72 h, followed by analysis using a CellTiter-Glo assay kit (Promega, Madison, WI, USA), according to the manufacturer's instructions.

### Flow cytometry

The cells were treated with indicated concentrations of GSK1904529A for 48 h and were subsequently harvested and stained with propidium iodide using a Cycletest Plus DNA reagent kit (BD Biosciences, Franklin Lakes, NJ, USA), followed by analysis of the DNA content using a FACSCalibur (BD Biosciences) and CellQuest Pro software version 5.1 (BD Biosciences).

### Apoptosis assay

Tumor samples, resected from mice, were fixed with fresh 10% formaldehyde and embedded into paraffin blocks. Cryosections were then prepared using a cryostat (CM1100; Leica Biosystems, Milton Keynes, UK). For terminal deoxynucleotidyl transferase dUTP nick end labeling (TUNEL) staining, the *in situ* cell death detection kit, TMR red (Roche Diagnostics, Madison, WI, USA) was used, according to the manufacturer's instructions. The nuclei were stained using Hoechst (Invitrogen Life Technologies, Carlsbad, CA, USA) for 20 min. Images were then captured using a fluorescent microscope (TE2000-E; Nikon Instruments, Melville, NY, USA). The animal experiments were approved by the Institutional Animal Care and Use Committee of Zhengzhou University (Zhengzhou, China).

The article "GSK1904529A, an insulin-like growth factor-1 receptor inhibitor, inhibits glioma tumor growth, induces apoptosis and inhibits migration" was published in 2015. Journal: Mol Med Rep.

### Transwell migration assay

A total of 1×10^5^ cells were seeded into the upper chamber of a 24-transwell Boyden chamber wells (Corning Incorporated, Corning, NY, USA) in serum-free complete DMEM in the absence or presence of various concentrations of GSK1904529A. Serum-free complete DMEM, supplemented with 20 *µ*g/ml fibronectin, was added to the lower chambers and used as a chemoattractant. The cells were treated with the indicated concentrations of GSK1904529A for 8 h and were subsequently fixed and stained using 0.1% crystal violet. The non-migrating cells on the upper chambers were removed and images of the migrated cells on the lower chambers were captured using a microscope in at least five randomly selected fields. The number of migrated cells were quantified and the inhibition of migration was calculated against the control group (no drug treatment).

### In vivo tumor investigation

A total of 2×10^6^ U87MG cells were implanted subcutaneously into the axillary flank of 16 female Balb/cA-nu mice aged 6–8 week (Shanghai Experimental Animal Center, Chinese Academy of Sciences, Shanghai, China). The animals were reared in a standard clean mouse facility. When the tumors reached 70 mm^3^ in size, the mice were randomly divided into a control group and GSK1904529A-treatment groups (6 mice/group). The mice in the GSK1904529A-treatment group received either 10 or 20 mg/kg GSK1904529A daily, and the control group received the same volume of vehicle control. The tumor volumes and body weights of the mice were measured daily. The tumor volume was calculated according to the following formula: (mm^3^) = 0.5 × (width × width × length).

### Statistical analysis

The measurement results of tumors in the drug treatment groups were compared with those of the control group (no drug treatment) at each time point and unpaired Student's t-test was used for the comparison of each time point. Statistical analysis was performed using SPSS 13.0 software (SPSS Inc., Chicago, IL, USA). The differences between each drug treatment group (10 and 20 mg/kg) and the control were statistically significant (P<0.05) for day 7, day 9 and day 11. P<0.05 was considered to indicate a statistically significant difference.

The article "GSK1904529A, an insulin-like growth factor-1 receptor inhibitor, inhibits glioma tumor growth, induces apoptosis and inhibits migration" was published in 2015. Journal: Mol Med Rep.

## Results

### GSK1904529A suppresses glioma cell viability

IGF/IGF-1R signaling contributes to the growth and survival of tumor cells (10). Therefore, the present study examined the effect of GSK1904529A on glioma cell viability. U87MG cells, commonly used human glioblastoma cells, were treated with increased concentrations of GSK1904529A and cell viability was determined. The data demonstrated that GSK1904529A significantly reduced the viability of U87MG cells in a dose-dependent manner, with a half-maximal inhibitory concentration (IC_50_) of ~50 nM (Fig. 1A). This suppression also increased as the duration of incubation increased (Fig. 1B). These data suggested that the U87MG cells were highly sensitive to inhibition by GSK1904529A.

### GSK1904529A induces the apoptosis of glioma cells

IGF/IGF-1R signaling has been demonstrated to protect cells from apoptosis (16). The present study examined the effect of GSK1904529A on the apoptosis of glioma cells. The U87MG cells were treated with increasing concentrations of GSK1904529A. The sub-G1 DNA content was determined using flow cytometry and was used to measure apoptosis. The data revealed that treatment with GSK1904529A significantly increased the sub-G1 DNA content in a dose-dependent manner (Fig. 2A). To confirm that apoptosis was induced by GSK1904529A, Hoechst staining was performed. The GSK1904529A-treated U87MG cells exhibited condensed and fragmented nuclei (Fig. 2B). The number of cells with an apoptotic morphology increased in a dose-dependent manner (Fig. 2C). Taken together, these data suggested that GSK1904529A markedly induced the apoptosis of glioma cells.

### GSK1904529A inhibits the migration of glioma cells

Glioma is a highly diffusely infiltrative disease. Motility is an important process, which contributes to glioma cell infiltration. It has been demonstrated that IGF/IGF-1R signaling stimulates motility in malignant cells (17). Therefore, the present study determined the effect of GSK1904529A on glioma cell migration. A Transwell migration assay was performed in the presence of increasing concentrations of GSK1904529A. As shown in Fig. 3A and B, the migration of the U87MG cells was significantly inhibited by treatment with GSK1904529A, and the inhibition occurred in a dose-dependent manner. These data suggested that GSK1904529A antagonized IGF/IGF-1R-stimulated glioma cell motility.

### GSK1904529A suppresses glioma tumor growth in vivo

As the present study demonstrated that GSK1904529A exhibited antitumor activity *in vitro*, the effect of GSK1904529A on tumor growth *in vivo* was determined. The U87MG cells were inoculated subcutaneously into the axillary regions of mice. Following tumor establishment, the mice were treated with GSK1904529A or vehicle control and the tumor volume was monitored. The data revealed that the mice treated with GSK1904529A exhibited substantially reduced tumor volumes compared with the vehicle-treated group (Fig. 4A). The suppression of tumor growth was correlated with the dose of GSK1904529A (Fig. 4A). In addition, the treatment was well tolerated, as no weight loss was observed (Fig. 4B). Further investigation revealed that treatment with GSK1904529A induced marked apoptosis in the tumor cells (Fig. 4C), which was consistent with the *in vitro* data. Taken together, these data suggested that GSK1904529A markedly inhibited glioma tumor growth *in vivo*.

The article "GSK1904529A, an insulin-like growth factor-1 receptor inhibitor, inhibits glioma tumor growth, induces apoptosis and inhibits migration" was published in 2015. Journal: Mol Med Rep.

## Discussion

Malignant gliomas have a particularly poor prognosis and is, therefore, a disease of significant concern. Efforts have been made to develop novel compounds and chemotherapeutics, however, these are focused on a limited number of targets, including epidermal growth factor receptor (EGFR) and platelet-derived growth factor receptor (PDGFR) (18). IGF/IGF-1R signaling has been implicated in malignant gliomas, suggesting it a potential therapeutic target. IGF antisense therapies are currently under evaluation in clinical trials (10). In the present study, the antitumor activity of a small-molecule inhibitor of IGF-1R, GSK1904529A, in glioma was assessed. The results demonstrated that GSK1904529A inhibited tumor growth *in vitro* and *in vivo* by inducing tumor cell apoptosis and inhibiting tumor cell migration. These results suggested that GSK1904529A is an effective compound for targeting IGF-1R and for the treatment of malignant gliomas.

Gliomas are a type of brain tumor, and the presence of the blood-brain barrier increases the difficulty for chemotherapeutic drugs to access the tumor. Further physiological investigations are required by introducing tumors into the brain to further assess the efficacy of GSK1904529A in the treatment of gliomas. With the development of increasing numbers of chemotherapeutic compounds, the combined therapy of GSK1904529A with other compounds may also be evaluated in the future studies.

In conclusion, the present study suggested the importance of the IGF/IGF-1R signaling pathway for the treatment of glioma. In addition, the results indicated that GSK1904529A may be a promising candidate for the treatment of glioma.

## Figures and Tables

**Figure 1:** GSK1904529A suppresses glioma cell viability. (A) U87MG cells were treated with GSK1904529A (6.25–400 nM) for 72 h, followed by measurement of cell viability using a viability assay. (B) U87MG cells were treated with GSK1904529A (100 nM) for 24, 48 or 72 h, followed by measurement of the effects on the inhibition of viability. Data are expressed as the mean ± standard deviation.

The article "GSK1904529A, an insulin-like growth factor-1 receptor inhibitor, inhibits glioma tumor growth, induces apoptosis and inhibits migration" was published in 2015. Journal: Mol Med Rep.

**Figure 2:** GSK1904529A induces apoptosis of glioma cells. (A) U87MG cells were treated with GSK1904529A at the indicated concentrations for 48 h, followed by staining with propidium iodide and flow cytometric analysis. (B) U87MG cells were incubated with 400 nM GSK1904529A for 48 h. The nuclei were stained using Hoechst and analyzed using a fluorescent microscope (magnification, x10). Representative images are shown. (C) Percentages of cells with condensed/fragmented nuclei were quantified in seven randomly selected fields. Data are expressed as the mean ± standard deviation.

**Figure 3:** GSK1904529A inhibits the migration of glioma cells. (A) U87MG cells were treated with GSK1904529A (10, 20 or 40 nM) for 8 h. The non-migrated cells on the upper surface of the filter were removed. The migrated cells on the lower surface were stained using crystal violet and images were captured (magnification, x4). Representative images are shown. (B) Quantification of the inhibition of Transwell migration. Data are expressed as the mean ± standard deviation.

**Figure 4:** GSK1904529A suppresses glioma tumor growth *in vivo*. (A) Following inoculation of the U87MG cells, GSK1904529A (10 or 20 mg/kg) was administered to the mice daily. The tumor volumes were measured every other day. (B) GSK1904529A (10 and 20 mg/kg) had no significant cytotoxic effects on the body weight of the mice during the treatments. (C) GSK1904529A (10 and 20 mg/kg) induced apoptosis of the U87MG tumor cells *in vivo*, measured using a TUNEL assay (green) and the nuclei were stained with Hoechst (blue; magnification, x4). TUNEL, terminal deoxynucleotidyl transferase dUTP nick end labeling. Data are expressed as the mean ± standard deviation.

## References

[1] Dolecek TA, Propp JM, Stroup NE, Kruchko C (2012). CBTRUS statistical report: Primary brain and central nervous system tumors diagnosed in the United States in 2005–2009. Neuro Oncol.

[2] Louis DN, Ohgaki H, Wiestler OD, Cavenee WK, Burger PC, Jouvet A, Scheithauer BW, Kleihues P (2007). The 2007 WHO classification of tumours of the central nervous system. Acta Neuropathol.

[3] Wen PY, Kesari S (2008). Malignant gliomas in adults. N Engl J Med.

[4] Omuro A, DeAngelis LM (2013). Glioblastoma and other malignant gliomas: A clinical review. JAMA.

[5] Anton K, Baehring JM, Mayer T (2012). Glioblastoma multiforme: Overview of current treatment and future perspectives. Hematol Oncol Clin North Am.

The article "GSK1904529A, an insulin-like growth factor-1 receptor inhibitor, inhibits glioma tumor growth, induces apoptosis and inhibits migration" was published in 2015. Journal: Mol Med Rep.

[6] Tognon CE, Sorensen PH (2012). Targeting the insulin-like growth factor 1 receptor (IGF1R) signaling pathway for cancer therapy. Expert Opin Ther Targets.

[7] Maki RG (2010). Small is beautiful: Insulin-like growth factors and their role in growth, development and cancer. J Clin Oncol.

[8] Miller BS, Yee D (2005). Type I insulin-like growth factor receptor as a therapeutic target in cancer. Cancer Res.

[9] Wang Y, Sun Y (2002). Insulin-like growth factor receptor-1 as an anti-cancer target: Blocking transformation and inducing apoptosis. Curr Cancer Drug Targets.

[10] Trojan J, Cloix JF, Ardourel MY, Chatel M, Anthony DD (2007). Insulin-like growth factor type I biology and targeting in malignant gliomas. Neuroscience.

[11] Resnicoff M, Sell C, Rubini M, Coppola D, Ambrose D, Baserga R, Rubin R (1994). Rat glioblastoma cells expressing an antisense RNA to the insulin-like growth factor-1 (IGF-1) receptor are nontumorigenic and induce regression of wild-type tumors. Cancer Res.

[12] Hägerstrand D, Lindh MB, Peña C, Garcia-Echeverria C, Nistér M, Hofmann F, Ostman A (2010). PI3K/PTEN/Akt pathway status affects the sensitivity of high-grade glioma cell cultures to the insulin-like growth factor-1 receptor inhibitor NVP-AEW541. Neuro Oncol.

[13] Bielen A, Perryman L, Box GM, Valenti M, de Haven Brandon A, Martins V, Jury A, Popov S, Gowan S, Jeay S (2011). Enhanced efficacy of IGF1R inhibition in pediatric glioblastoma by combinatorial targeting of PDGFRα/β. Mol Cancer Ther.

[14] Shi ZM, Wang XF, Qian X, Tao T, Wang L, Chen QD, Wang XR, Cao L, Wang YY, Zhang JX, Jiang T (2013). MiRNA-181b suppresses IGF-1R and functions as a tumor suppressor gene in gliomas. RNA.

[15] Sabbatini P, Rowand JL, Groy A, Korenchuk S, Liu Q, Atkins C, Dumble M, Yang J, Anderson K, Wilson BJ (2009). Antitumor activity of GSK1904529A, a small-molecule inhibitor of the insulin-like growth factor-I receptor tyrosine kinase. Clin Cancer Res.

[16] Peruzzi F, Prisco M, Dews M, Salomoni P, Grassilli E, Romano G, Calabretta B, Baserga R (1999). Multiple signaling pathways of the insulin-like growth factor 1 receptor in protection from apoptosis. Mol Cell Biol.

[17] Meyer GE, Shelden E, Kim B, Feldman EL (2001). Insulin-like growth factor I stimulates motility in human neuroblastoma cells. Oncogene.

[18] Prabhu S, Harris F, Lea R, Snape TJ (2014). Small-molecule clinical trial candidates for the treatment of glioma. Drug Discov Today.

